The article "The promises and challenges of AI-based chatbots in language education through the lens of learner emotions" was retracted in 2025. Reasons: unreliable results or conclusions; concerns about the citations.

# The promises and challenges of AI-based chatbots in language education through the lens of learner emotions

**DOI:** 10.1016/j.heliyon.2024.e37238

**Published:** 2024-09-03

**Authors:** Yuehai Xiao, Tianyu Zhang, Jingyi He

**Affiliations:** Department of English, Hunan Normal University, Changsha City, China

**Keywords:** AI-based chatbots, Language education, Positive psychology, Learner emotions, Chatbot-learner interactions

## Abstract

The integration of AI-based chatbots in language education has garnered significant attention, yet the interplay between chatbots and positive psychology remains underexplored. Filling this gap through a critical analysis of existing theories, measurement scales, and empirical evidence, this paper evaluates the potential benefits and drawbacks of incorporating AI chatbots in language learning environments and how AI chatbots may positively or negatively impact emotional dimensions of language acquisition. The findings unravel that the primary advantages of the AI chatbots are personalized instruction with rapid feedback, a decrease in anxiety levels and a surge in motivation, greater learner independence and self-directed learning, and the fostering of metacognitive abilities. Conversely, the identified obstacles encompass restricted emotional awareness, a deficiency in genuine human interaction, ethical dilemmas and privacy issues, as well as the potential reinforcement of biases and stereotypes. By highlighting the importance of learner emotions in the language learning process, this conceptual analysis review underscores the need for a nuanced understanding of how AI chatbots can support or hinder emotional engagement and motivation. The paper discusses the impacting factors of AI-based chatbots in language education, and strategies for addressing challenges and optimizing chatbot-learner interactions, such as incorporating affective computing techniques and designing culturally-sensitive chatbots. Finally, the article outlines future research directions, emphasizing the need for validated emotion scales in chatbot assisted language learning contexts, longitudinal studies, mixed-methods research, comparative analyses, and investigations into the role of chatbots in fostering emotional intelligence and intercultural competence.

## Highlights

• AI chatbots' impact on learner emotions in language education explored.
• Empirical studies and theories synthesized for chatbot benefits and challenges.
• Calling for new scales to measure learner emotions in the context of chatbot-assisted language learning.
• The factors affecting learner emotions in using chatbots in language education.
• Promises and challenges of AI-based chatbots in language education.

## 1 Introduction

The rapid advancement of artificial intelligence (AI) has led to the development of chatbots, such as ChatGPT-4o and Claude 3, which are increasingly being utilized in various educational contexts, including language learning [[1], [2], [3], [4], [5]]. AI-based chatbots offer several affordances in language education, such as providing personalized and interactive learning experiences, increasing learner engagement, and offering 24/7 availability [4,6]. However, the use of chatbots in language learning has also sparked controversies, raising concerns about privacy, data security, and the potential for chatbots to replace human teachers [7].

Another growing body of literature concerns positive psychology, including learner emotions, which play a crucial role in the language learning process, influencing factors such as motivation, engagement, and academic achievement [8]. Positive emotions, such as enjoyment, motivation, grit, self-efficacy, patience, engagement, emotion regulation, loving pedagogy, growth mindset, and empathy, foster a supportive learning environment, encourage risk-taking, and promote resilience in the face of challenges [9,10]. Conversely, negative emotions, including anxiety, fear, anger, demotivation, disengagement, boredom, and burnout, may cause learners to avoid participation and risk-taking, with negative attitudes towards language learning [11,12]. As AI-based chatbots become increasingly prevalent in language education, it is essential to consider how these technologies can be designed and implemented to cultivate positive emotions and mitigate the impact of negative emotions on learners' experiences and outcomes.

These chatbots, powered by sophisticated algorithms, are designed to interact with learners in a conversational manner, providing instant feedback and personalized learning paths [13]. A notable example is the use of the AI chatbot “Ellie," which has been implemented to assist in language learning by offering empathetic responses and adapting to the learner's emotional state [14]. Another instance is the application of “ChatGPT," which has been utilized in educational settings to facilitate English language learning, including vocabulary acquisition and pronunciation practice [15].

Preliminary findings suggest that AI chatbots have a significant impact on learner emotions. For instance, research indicates that AI chatbots can reduce language learning anxiety by providing a low-pressure environment for practice, where learners can converse freely without the fear of judgment [16]. This reduction in anxiety is crucial, as it allows learners to engage more actively in language practice, leading to improved language proficiency and communication skills [13]. Additionally, the interactive and adaptive nature of AI chatbots can enhance learner motivation, as they offer a sense of companionship and personalized feedback that caters to individual learning needs [14].

However, challenges persist. Technical limitations, such as the inability of some chatbots to understand complex expressions or provide nuanced feedback, can lead to learner frustration and disengagement [15]. Furthermore, concerns about data privacy and the potential for AI chatbots to replace human teachers also influence learner emotions and perceptions of the learning experience [16].

To sum up, as AI chatbots become more prevalent in language education, it is imperative to consider their emotional impact on learners. While they offer promising benefits in terms of accessibility, personalization, and engagement, addressing the challenges related to emotional design and technological limitations will be crucial for optimizing their effectiveness in language learning contexts. As such, there is a need for a critical analysis that examines the promises and challenges of AI-based chatbots in language education through the lens of learner emotions.

This review article serves multiple interconnected aims that enhance our understanding of the integration of AI chatbots to language learning and the potential impact on learner emotions.

As Table 1 illustrates, the purpose and scope of this article encompass the following: To critically evaluate the current landscape of AI-based chatbots in language education; To explore the theoretical underpinnings that support the use of chatbots in language learning contexts; To review existing measurement scales that quantify the emotional impact on learners; To analyze the affordances and controversies that chatbots introduce to language education; To review empirical studies that provide evidence of the influence of chatbots on learner emotions; To consider a wide scope that encompasses various language learning contexts, including formal education, self-directed learning, and supplementary language instruction.

**Table 1:** Purposes and scope of the review article.

No.	
1	Critical evaluation of AI chatbots in language education
2	Exploration of theoretical underpinnings
3	Review of measurement scales for emotional impact
4	Analysis of affordances and controversies
5	Review of empirical studies on influence on emotions
6	Consideration of various language learning contexts
7	Highlighting the importance of learner emotions
8	Offering interdisciplinary insights

The chatbot-emotion relationship, while showing promise, remains an underexplored territory, particularly in understanding the nuanced interplay between chatbot design features and the wide spectrum of emotional outcomes they can elicit in educational settings. Current research in the existing literature has just begun to scratch the surface regarding how chatbots' empathy, cultural sensitivity, and adaptive learning capabilities can influence learners' emotional experiences and, in turn, their cognitive engagement and academic performance. There is a pressing need for more investigation into how chatbots can be tailored to support diverse emotional needs, especially for students with different learning styles, backgrounds, or those facing socio-emotional challenges. This conceptual analysis paper aims to underscore these issues, highlighting the practical relevance and potential impact of further research in this burgeoning field.

This review article, as summarized in Table 2, makes the following key contributions:

1. It underscores the benefits of AI chatbots in language learning, including personalized instruction, immediate feedback, and reduction of language anxiety.
2. It addresses the challenges, such as technical limitations, privacy issues, and emotional disconnection in AI interactions.
3. It stresses the necessity of accounting for learners' emotions in AI chatbot design for language education.
4. It integrates empirical research, theoretical insights, and practical applications for a holistic perspective on AI chatbots.
5. It advises educators on integrating AI chatbots into language teaching, considering emotional aspects.
6. It guides policymakers in establishing frameworks for the ethical use of AI in education.
7. It suggests directions for future research to bridge knowledge gaps, particularly in long-term emotional impacts and varied learning contexts.
8. It tracks the advancement of AI chatbots in language education, emphasizing emotional intelligence and engagement.

**Table 2:** Main contributions of this article.

No.	
1	Highlighting the positive aspects of AI chatbots
2	Discussion of the challenges faced
3	Emphasis on a learner-centered approach
4	Provision of interdisciplinary insights
5	Offering pedagogical implications for educators
6	Providing policy recommendations for stakeholders
7	Proposing areas for future research
8	Monitoring technological advancements in AI chatbots

This review paper aims to be a pivotal contribution to the field, offering a nuanced perspective on the intersection of AI chatbots, and language education, with a spotlight on the emotional well-being of learners. Through this multifaceted approach, the article seeks to inform and inspire stakeholders to make informed decisions about the integration of AI chatbots in language learning ecosystems.

## 2 Literature review

### 2.1 Theoretical frameworks

The integration of AI-based chatbots in language education can be understood through various theoretical lenses. One prominent theory is the Connectivism learning theory, which emphasizes the role of technology in facilitating learning in the digital age [17]. According to Connectivism, learning occurs through the formation of connections between information sources, and technology plays a crucial role in enabling these connections. AI-based chatbots, as a form of educational technology, can be seen as a means of facilitating learning by providing learners with personalized, interactive, and readily accessible language learning experiences [18].

Another relevant theory is the Interaction Hypothesis, which posits that language acquisition occurs through meaningful interactions between learners and interlocutors [19]. AI-based chatbots can serve as interactive partners for language learners, providing opportunities for learners to engage in meaningful language exchanges and negotiate meaning [3,4,6]. However, the quality and authenticity of these interactions may be limited by the chatbots' artificial nature, highlighting the need for further research on the effectiveness of chatbot-learner interactions in promoting language acquisition.

Positive psychology is a field that investigates the factors contributing to human flourishing and well-being [20]. Within this broader framework, the Control-Value Theory provides a lens through which to examine the emotional experiences of learners engaging with AI-based chatbots in language education.

The Control-Value Theory posits that learners' emotions are influenced by their perceived control over learning activities and outcomes, as well as the subjective value they attach to these activities and outcomes [21]. According to this theory, learners experience positive emotions, such as enjoyment and pride, when they perceive high levels of control and value in their learning experiences. Conversely, learners may experience negative emotions, such as anxiety and frustration, when they perceive low levels of control and value [22].

In the context of AI-based chatbots in language education, the Control-Value Theory provides a valuable framework for understanding how learners' emotional experiences may be shaped by their interactions with these technologies. For example, chatbots that are designed to provide learners with a sense of autonomy and control over their learning process may foster positive emotions and enhance motivation [23]. On the other hand, chatbots that are perceived as inflexible or unresponsive to learners' needs may lead to negative emotional experiences and hinder learning [24].

Furthermore, the perceived value of AI-based chatbots in language education may also influence learners' emotional experiences. Chatbots that are seen as providing meaningful and relevant learning opportunities are more likely to elicit positive emotions and engagement from learners [2]. In contrast, chatbots that are viewed as trivial or disconnected from learners' goals and interests may lead to disengagement and negative emotions.

By examining the promises and challenges of AI-based chatbots in language education through the lens of the Control-Value Theory, this conceptual article aims to provide a nuanced understanding of how these technologies can be designed and implemented to optimize learners' emotional experiences and, ultimately, their language learning outcomes. The insights gained from this theoretical perspective will contribute to the growing body of knowledge on the affective dimensions of technology-enhanced language learning and inform future research and practice in this field.

Another positive psychology theory that provides a valuable framework for understanding the role of learner emotions in language education and how AI-based chatbots can influence these emotions is the Broaden-and-Build Theory of Positive Emotions [25]. According to this theory, positive emotions broaden an individual's thought-action repertoire, leading to increased creativity, exploration, and personal growth. In the context of language learning, positive emotions experienced during interactions with chatbots can encourage learners to engage more actively, take risks, and explore the language in novel ways [26]. This broadened perspective can foster a growth mindset, where learners view challenges as opportunities for learning and development [8]. Moreover, the positive emotions generated through chatbot interactions can build learners' psychological resources, such as resilience, self-efficacy, and social connections, which contribute to long-term language learning success and well-being [27]. By designing chatbots that prioritize the cultivation of positive emotions, language educators can create a supportive and engaging learning environment that promotes learners' personal and linguistic growth.

Self-Determination Theory [28] is the third relevant positive psychology theory, which emphasizes the importance of autonomy, competence, and relatedness in fostering intrinsic motivation. AI-based chatbots can support learner autonomy by providing personalized learning experiences and allowing learners to control the pace and content of their interactions. Chatbots can also contribute to learners' sense of competence by offering scaffolded support and adaptive feedback. However, the extent to which chatbots can satisfy learners' need for relatedness may be limited, as the emotional connection between learners and chatbots may not be as strong as that between learners and human teachers [5].

The theoretical framework presented here will guide the analysis and synthesis of existing research, helping to identify gaps in the literature and provide directions for future research and practice. This conceptual article aims to provide a comprehensive understanding of how chatbots can influence learner emotions and, consequently, language learning outcomes. This paper calls for more research to examine the promises and challenges of AI-based chatbots in language education through the lenses of connectivism, interaction hypothesis, and positive psychology theories.

### 2.2 How do the theoretical frameworks complement and intersect

In the context of AI-based chatbots in language education, particularly regarding learners' emotions, the above mentioned theoretical frameworks complement and intersect in various ways:

1. Connectivism and Interaction Hypothesis: Connectivism, which emphasizes the role of technology in creating a networked learning environment, intersects with the interaction hypothesis by suggesting that AI chatbots can facilitate meaningful interactions necessary for language acquisition. Chatbots can simulate conversations, providing learners with opportunities to practice language skills in a digital environment.
2. Positive Psychology Theories and Broaden-and-Build Theory: Positive psychology theories focus on human flourishing, which can be enhanced through the broaden-and-build theory of positive emotions. In language learning, AI chatbots can be designed to provide positive feedback and encouragement, fostering a positive emotional state that broadens learners' thinking and enhances creativity and exploration in language use.
3. Control-Value Theory and Self-Determination Theory: Both theories intersect in the context of learner autonomy. AI chatbots can be programmed to adapt to individual learner needs, providing a sense of control over the learning process, which is central to the control-value theory. This autonomy, combined with a chatbot's ability to affirm the value of learning activities, can also address the needs for competence and relatedness as outlined in self-determination theory, thereby increasing intrinsic motivation.
4. Interaction Hypothesis and Self-Determination Theory: The interaction hypothesis can be enriched by self-determination theory's emphasis on the importance of social interaction. Meaningful interactions facilitated by chatbots can not only lead to language acquisition but also satisfy learners' need for relatedness, a key component of intrinsic motivation.
5. Connectivism and Broaden-and-Build Theory: Connectivism's focus on technology-enabled learning networks can be expanded by the broaden-and-build theory's assertion that positive emotions lead to personal growth. The interconnectedness of digital learning can provide a platform for diverse interactions, which, when positive, can broaden learners' horizons and build their capacities.
6. Control-Value Theory and Interaction Hypothesis: The perceived control learners have over chatbot-assisted learning activities, as posited by control-value theory, can influence the quality of interactions. When learners feel in control of the interaction pace and content, it may lead to more meaningful and effective language practice, in line with the interaction hypothesis.
7. Positive Psychology Theories and Self-Determination Theory: Both theories recognize the importance of internal factors in motivation. Positive psychology focuses on well-being and flourishing, while self-determination theory highlights autonomy, competence, and relatedness. When AI chatbots are designed with these principles in mind, they can contribute to a learning environment that promotes intrinsic motivation and a positive emotional state.
8. Self-Determination Theory and Broaden-and-Build Theory: The satisfaction of psychological needs as described by self-determination theory can lead to positive emotions, which, according to the broaden-and-build theory, can enhance learners' capabilities and resilience. AI chatbots can be programmed to support learners' psychological needs, fostering an environment conducive to positive emotional outcomes.

In summary, these theories provide a comprehensive framework for understanding how AI chatbots can be leveraged to enhance language learning by considering learners' emotional experiences. The intersection of these theories suggests that AI chatbots, when designed with empathy for learners' emotional needs and motivational factors, can create a supportive and effective language learning environment.

Below are some conceptual examples of how Connectivism, Interaction Hypothesis, and positive psychology might be applied in AI-based chatbots for language education:

1. Connectivism in AI Chatbots: Connectivism posits that learning is a networked process, facilitated by connections within a digital ecosystem. An AI chatbot could be designed to connect learners with various language learning resources, such as online dictionaries, pronunciation guides, and cultural notes. For instance, a chatbot might offer links to videos or articles that provide context for language use, thus enhancing the learning experience through a network of information [17].
2. Interaction Hypothesis with AI Chatbots: According to the Interaction Hypothesis, language acquisition is optimized through interaction that involves negotiation of meaning. An AI chatbot could simulate conversational partners for learners, providing immediate feedback and corrections, which is crucial for language learning [29]. For example, a chatbot might engage a learner in a role-play scenario, offering responses that prompt the learner to use new vocabulary or grammar structures.
3. Positive Psychology in AI Chatbots: Positive psychology focuses on promoting well-being and personal strengths. An AI chatbot could incorporate elements of positive psychology by recognizing and praising learners' achievements, providing motivational messages, and setting achievable goals that boost learners' confidence and intrinsic motivation [30]. For example, a chatbot might use phrases like “Great job! You're improving your vocabulary," to reinforce positive learning outcomes.

### 2.3 How can AI chatbots affect learner emotions

AI-based chatbots can influence learner emotions in various ways, and positive psychology theories provide a framework for understanding these impacts.

Below is Table 3 about how AI chatbots can affect learner emotions:

**Table 3:** How AI chatbots affect learner emotions.

No.	Aspect of AI Chatbots	Influence on Learner Emotions	Theoretical Framework	Supporting Evidence
1	Immediate Feedback	Reinforces confidence, reduces anxiety	Broaden-and-Build Theory	[31]
2	Personalization	Enhances autonomy, competence, relatedness	Self-Determination Theory	[32]
3	Availability	Reduces isolation, increases support	N/A	N/A
4	Safety of Practice	Lowers inhibitions, reduces fear of mistakes	N/A	[33,34]
5	Engagement	Increases motivation through gamified elements	Self-Determination Theory	[32]
6	Emotional Recognition	Provides empathetic responses, strengthens emotional connection	Positive Psychology	[30]
7	Reducing Cognitive Load	Alleviates stress from information overload	N/A	N/A
8	Cultural Sensitivity	Promotes inclusivity and positive emotional environment	N/A	N/A

Table 3 suggests that AI chatbots can affect learner emotions in the following ways:

1. Provision of Immediate Feedback: AI chatbots offer instant responses and feedback, which can reinforce learners' confidence and reduce anxiety associated with waiting for responses from human teachers [31]. Positive feedback from chatbots, aligned with the Broaden-and-Build Theory [25], can broaden learners' thought-action repertoires, encouraging creativity and exploration in language use.
2. Personalization and Adaptation: Chatbots can adapt to individual learner needs, which aligns with Self-Determination Theory's emphasis on autonomy [32]. Personalized learning paths can enhance learners' sense of competence and relatedness, fostering intrinsic motivation and a positive emotional state.
3. Availability and Accessibility: The availability of chatbots 24/7 can provide learners with a constant learning companion, reducing feelings of isolation and increasing a sense of support, which is crucial for emotional well-being and learning engagement.
4. Safety of Practice: The anonymity provided by interacting with a chatbot can lower inhibitions and reduce the fear of making mistakes, which is a significant source of anxiety for language learners. This safety net can help learners express themselves more freely, thus positively impacting their emotional state and willingness to engage with the language [33,34].
5. Engagement and Motivation: Gamified elements and interactive features of AI chatbots can make language learning more engaging and motivating. According to Self-Determination Theory, when learners feel autonomous and competent, they are more likely to experience positive emotions and enjoy the learning process [32].
6. Emotional Recognition and Responsiveness: Advanced AI chatbots capable of recognizing and responding to learners' emotions can provide an empathetic learning environment. This emotional intelligence can lead to a stronger emotional connection between the learner and the chatbot, which is in line with positive psychology's focus on emotional well-being contributing to overall flourishing [30].
7. Reducing Cognitive Load: By providing clear, concise information and explanations, chatbots can reduce cognitive load, allowing learners to focus on language acquisition without the stress of information overload, which can negatively impact emotions.
8. Cultural Sensitivity: AI chatbots can be programmed to be culturally sensitive, acknowledging and adapting to the diverse emotional expressions and communication preferences of learners from different backgrounds, thus promoting a positive and inclusive learning environment.

It's important to note that while positive psychology theories provide a lens to understand the potential positive impacts of AI chatbots on learner emotions, empirical research is necessary to validate these theoretical perspectives in practical educational settings.

### 2.4 Calling for developing new scales to measure learner emotions in using chatbots in language education

Learner emotions play a crucial role in the language learning process, and the emergence of AI-based chatbots in language education has prompted us to call for more research to investigate the emotional experiences of learners when interacting with these tools. To measure learner emotions in the context of chatbot-assisted language learning, various scales need to be developed, validated and employed in studies pertain to the interplay between chatbots and language learner emotions. Positive emotions, such as enjoyment, motivation, grit, self-efficacy, patience, engagement, emotion regulation, loving pedagogy, growth mindset, and empathy, have been identified as essential factors in successful language learning (see also [35]).

Measuring language learners' positive emotions has been a crucial aspect of understanding their learning experiences and outcomes. Several scales have been employed by researchers to assess these emotions, including Academic Grit Scale [36] and the Positive and Negative Affect Schedule (PANAS) [37]. The Foreign Language Enjoyment Scale, developed by Dewaele and MacIntyre [38] and further validated by Botes et al. [39], is a psychometric instrument specifically designed to measure foreign language learners' enjoyment. Additionally, the construct of grit, defined as perseverance and passion for long-term goals, has been measured using the Grit Scale [40] and the Metacognitive Awareness of Grit Scale (MCAGS) [41]. These scales have provided valuable insights into the role of positive emotions and grit in language learning, and their application in the context of AI-based chatbots could shed light on how these technologies influence learners' emotional experiences and learning outcomes.

More researchers may adapt existing scales to measure these emotions in the context of chatbot-assisted language learning. For example, the Foreign Language Enjoyment Scale [38] can be modified to assess learners' enjoyment when interacting with chatbots. Similarly, the Motivated Strategies for Learning Questionnaire [42] can be adapted to measure learners' motivation and self-efficacy in chatbot-based language learning environments.

Furthermore, there is a scarcity of new scales specifically designed to measure positive emotions in the context of chatbot-assisted language learning. This highlights the need for the development and validation of new scales that capture the unique emotional experiences of learners when interacting with AI-based chatbots. Such scales should consider the specific affordances and limitations of chatbots, as well as the potential impact of chatbot design features on learner emotions.

Negative emotions, such as anxiety, fear, anger, demotivation, disengagement, boredom, and burnout, can hinder language learning progress and lead to poor performance [11]. Researchers may investigate the presence of these negative emotions in chatbot-assisted language learning, as the use of standardized scales to measure these emotions has been limited. For instance, the Foreign Language Classroom Anxiety Scale and Foreign Language Boredom Scale [43] can be adapted to assess learners' anxiety and boredom when interacting with chatbots. Furthermore, the unique characteristics of chatbot-based interactions may require the development of new scales that specifically address the potential sources of negative emotions in this context, such as the lack of human-like empathy or the frustration arising from technical limitations.

Future research should focus on creating new scales that assess positive and negative emotions, taking into account the specific affordances and limitations of AI-based chatbots in language education. Such scales will provide valuable insights into the emotional dimensions of chatbot-assisted language learning and inform the design and implementation of emotionally intelligent chatbots that promote positive learning experiences.

### 2.5 The factors affecting learner emotions in using chatbots in language education

Numerous factors may impact learner emotions in chatbot-assistedlanguagelearning, encompassing access to chatbots, learners' AI literacy, the user interface design of chatbots, personalization and adaptation, how chatbots handle errors and provide feedback, the natural language processing (NLP) capabilities of chatbots, and cultural factors.

Access to AI technology, particularly chatbots, can significantly impact learner emotions in language education. When learners have limited access to chatbots, they may experience frustration or a sense of exclusion from the learning experience. This digital divide can create emotional barriers that hinder language acquisition and overall engagement [44]. Learners who cannot access chatbots may feel disadvantaged compared to their peers who have the opportunity to benefit from this technology. On the other hand, when chatbots are widely accessible, learners are more likely to experience positive emotions such as excitement, curiosity, and a sense of inclusion [45]. Ensuring equitable access to chatbot technology is crucial for promoting positive learner emotions and creating an inclusive language learning environment. Learners' AI literacy, or their familiarity and comfort with using AI technology, can greatly influence their emotions when interacting with chatbots in language education. Learners with higher AI literacy tend to feel more confident and positive about using chatbots, as they understand the capabilities and limitations of the technology [46]. They are more likely to engage with chatbots effectively, leading to a more enjoyable and productive learning experience. In contrast, learners with lower AI literacy may experience anxiety, uncertainty, or even skepticism when using chatbots. They may struggle to navigate the technology or have unrealistic expectations, leading to frustration or disappointment [47]. Providing learners with adequate training and support to develop their AI literacy is essential for fostering positive emotions and ensuring a smooth adoption of chatbot technology in language education.

The user interface design of chatbots plays a crucial role in shaping learner emotions in language education. A well-designed, user-friendly, and intuitive interface can enhance positive emotions and facilitate a seamless learning experience. When learners can easily navigate and interact with the chatbot, they are more likely to feel engaged, motivated, and satisfied with the learning process [48]. On the other hand, a complex, confusing, or poorly designed interface can lead to frustration, irritation, and disengagement. Learners may struggle to find the information they need or become overwhelmed by the cognitive load required to use the chatbot effectively [49]. To promote positive learner emotions, it is essential for chatbot developers to prioritize user-centered design principles, conduct usability testing, and continuously iterate based on learner feedback. By creating intuitive and visually appealing interfaces, chatbots can foster a positive emotional experience and enhance language learning outcomes.

Personalization and adaptation play a vital role in shaping learner emotions when using chatbots in language education. Chatbots that can tailor their interactions to individual learners' needs, preferences, and abilities have the potential to enhance engagement and motivation. By providing personalized recommendations, feedback, and content that aligns with learners' interests and proficiency levels, chatbots can create a more meaningful and enjoyable learning experience [50]. This individualized approach can foster positive emotions such as satisfaction, confidence, and a sense of achievement. Moreover, adaptive chatbots that can adjust their language complexity and pace based on learners' performance can prevent frustration and maintain learner engagement [51]. The way chatbots handle errors and provide feedback can significantly influence learner emotions in language education. Effective error handling involves clear explanations, gentle correction, and constructive feedback that encourages learners to learn from their mistakes. When chatbots offer supportive and informative feedback, learners are more likely to experience positive emotions such as motivation and a sense of progress [52]. On the other hand, harsh, critical, or unhelpful feedback can lead to negative emotions like frustration, demotivation, and self-doubt. Chatbots that prioritize a supportive and nurturing approach to error correction can contribute to a positive learning environment that promotes emotional well-being and fosters language acquisition (Ramadan & Jember, 2024). The natural language processing (NLP) capabilities of chatbots can significantly impact learner emotions in language education. Chatbots with advanced NLP can understand and generate more accurate and meaningful responses, leading to a more engaging and satisfying learning experience. When chatbots can effectively interpret learners' input and provide relevant and coherent responses, learners are more likely to experience positive emotions such as enjoyment, curiosity, and a sense of accomplishment [53]. In contrast, chatbots with limited NLP capabilities may generate irrelevant or nonsensical responses, causing frustration and disengagement among learners. Therefore, the development of chatbots with robust NLP is crucial for fostering positive learner emotions and facilitating effective language learning [54]. Cultural factors play a significant role in shaping learner emotions when interacting with chatbots in language education. Chatbots that demonstrate cultural sensitivity, use appropriate language, and respect cultural norms can contribute to a positive and inclusive learning experience. By incorporating culturally relevant content and examples, chatbots can help learners feel more connected and engaged with the learning material [55]. Additionally, chatbots that avoid cultural stereotypes and promote diversity and inclusiveness can foster a sense of belonging and emotional well-being among learners from different cultural backgrounds. On the other hand, chatbots that lack cultural sensitivity or perpetuate stereotypes may lead to negative emotions such as alienation, discomfort, or even offense [56]. Therefore, it is essential for chatbots in language education to be designed with cultural considerations in mind to ensure a positive emotional experience for all learners. It's important to note that these factors may vary depending on individual learners and their specific contexts.

## 3 Findings

### 3.1 The promises of AI-based chatbots in language education

As Table 4 shows, first of all, AI-based chatbots in language education hold great promises in providing personalized learning experiences for learners. One of the key advantages of chatbots is their ability to adapt to learners' proficiency levels, ensuring that the content and interactions are tailored to each individual's needs [57]. By assessing learners' language skills and adjusting the complexity and pace of the learning material accordingly, chatbots can create a more effective and engaging learning environment [51]. Moreover, chatbots can cater to individual learning styles and preferences, offering a variety of activities and resources that align with learners' interests and preferred methods of learning [58]. This personalization not only enhances learning outcomes but also fosters positive emotions such as satisfaction, confidence, and motivation among learners.

**Table 4:** The promises of AI-Based chatbots in language education

No.	Promises of AI-Based Chatbots	Description of Impact
1	Personalized Learning	Chatbots adapt to learners' proficiency levels, offering tailored content and interactions, which enhances learning outcomes and fosters positive emotions such as satisfaction, confidence, and motivation.
2	Reduced Anxiety and Increased Motivation	Chatbots provide a non-judgmental learning environment, reducing anxiety and encouraging learners to take risks and learn from their mistakes, thus promoting a growth mindset and learner autonomy.
3	Enhanced Learner Autonomy and Self-Regulated Learning	By offering 24/7 access to language learning resources, chatbots empower learners to take control of their learning journey, allowing them to engage at their own pace and fit language learning into their routines.
4	Promotion of Metacognitive Skills	Through learner-initiated interactions and self-reflection with chatbots, learners develop a deeper understanding of their strengths, weaknesses, and learning strategies, leading to increased motivation, persistence, and a sense of accomplishment.

Secondly, chatbots in language education have the potential to reduce learner anxiety and increase motivation by providing a non-judgmental learning environment. Many language learners experience anxiety when practicing their skills in front of others, fearing mistakes or negative evaluations [59]. Chatbots offer a non-threatening environment where learners can practice without the fear of being judged or embarrassed. This low-stakes environment encourages learners to take risks, experiment with the language, and learn from their mistakes.

This supportive atmosphere fosters learner autonomy and promotes a growth mindset, as learners feel more comfortable exploring the language and learning from their experiences [60]. By providing a judgment-free zone for language practice, chatbots empower learners to take ownership of their learning and develop their communicative competence.

As a result, learners are more likely to experience positive emotions such as confidence, enjoyment, and a sense of progress. Moreover, chatbots can provide immediate feedback and encouragement, further boosting learner motivation and engagement [61]. Thirdly, AI-based chatbots have the potential to enhance learner autonomy and promote self-regulated learning in language education. By offering 24/7 access to language learning resources, chatbots empower learners to take control of their learning journey [62]. Learners can engage with the chatbot at their own pace, choosing when and how to practice their language skills. This flexibility allows learners to fit language learning into their daily routines and encourages them to take responsibility for their progress [63].

Fourthly, chatbots can promote learner-initiated interactions and self-reflection, fostering metacognitive skills. By engaging in meaningful conversations with the chatbot and reflecting on their performance, learners develop a deeper understanding of their strengths, weaknesses, and learning strategies [64]. This self-awareness and self-regulation can lead to increased motivation, persistence, and a sense of accomplishment, ultimately contributing to positive learner emotions and successful language acquisition.

### 3.2 The challenges of AI-based chatbots in language education

On the other hand, however, using chatbots in language learning may pose certain challenges.

Demonstrated by Table 5, one of the significant challenges of AI-based chatbots in language education is their limited emotional intelligence and empathy. While chatbots can provide personalized learning experiences, they may struggle to recognize and respond appropriately to learners' emotional states [65]. This limitation can lead to misunderstandings and a lack of emotional support, which are crucial for maintaining learner engagement and motivation [66]. For example, if a learner expresses frustration or confusion, a chatbot may not be able to offer the same level of empathy and reassurance as a human teacher. Moreover, chatbots may misinterpret learners' intentions and needs, leading to inappropriate or irrelevant responses that can negatively impact learner emotions [67]. Addressing these limitations in emotional intelligence and empathy is essential for creating a more supportive and emotionally attuned learning environment.

**Table 5:** The challenges of AI-Based chatbots in language education.

No.	Challenges of AI-Based Chatbots	Description of Challenge
1	Limited Emotional Intelligence	AI chatbots may struggle to recognize and respond to learners' emotional states, leading to a lack of emotional support crucial for engagement and motivation.
2	Lack of Authentic Human Interaction	Chatbots cannot fully replicate the richness of human communication, lacking non-verbal cues and potentially limiting the depth of language learning experiences.
3	Ethical Concerns and Data Privacy	Interactions with chatbots raise data privacy issues, requiring robust data protection measures and transparency about data usage.
4	Perpetuation of Biases and Stereotypes	Chatbot algorithms might perpetuate societal biases if trained on data reflecting inequalities or misconceptions, necessitating efforts to ensure equity and inclusion.

Another challenge of AI-based chatbots in language education is the lack of authentic human interaction and cultural context. While chatbots can simulate conversations and provide language practice opportunities, they cannot fully replicate the richness and complexity of human communication [68]. The absence of non-verbal cues, such as facial expressions, gestures, and tone of voice, can limit the depth and nuance of the learning experience. Moreover, chatbots may not be able to provide learners with sufficient exposure to real-life language use and cultural nuances (Belda & Kokošková, 2023). Language learning is not just about acquiring linguistic skills but also understanding the cultural context in which the language is used. Chatbots may struggle to convey the subtle cultural differences and social norms that are essential for effective communication in real-world situations [56]. Balancing chatbot-based learning with authentic human interaction and cultural immersion is crucial for fostering a well-rounded language education.

Thirdly, AI-based chatbots in language education also raise ethical concerns and data privacy issues that need to be addressed. As learners interact with chatbots, they may share personal information, such as their learning progress, preferences, and even sensitive data [69]. Protecting learners' privacy and ensuring the security of their data is of utmost importance. Educational institutions and chatbot developers must implement robust data protection measures and be transparent about how learners' information is collected, stored, and used [70]. Failure to prioritize data privacy and security can lead to breaches, unauthorized access, or misuse of learners' personal information, which may have severe consequences for their emotional well-being and willingness to engage with chatbots in language learning [7].

Finally, chatbot algorithms may inadvertently perpetuate biases and stereotypes, particularly when trained on data that reflects societal inequalities or cultural misconceptions [4,71]. For example, a chatbot may generate responses that are politically correct in the US context but may not be appropriate or inclusive in other cultural settings. Addressing these biases and ensuring that chatbots promote diversity, equity, and inclusion is a critical challenge that requires ongoing attention and effort from researchers, developers, and educators alike.

### 3.3 Strategies for addressing challenges and optimizing chatbot-learner interactions

To address the challenges related to learner emotions and empathy in AI-based chatbots, researchers and developers can incorporate affective computing and sentiment analysis techniques. Affective computing focuses on creating systems that can recognize, interpret, and respond to human emotions [50]. By integrating these techniques, chatbots can better detect learners' emotional states based on their language use, tone, and other cues. For example, sentiment analysis algorithms can analyze learners' responses and provide appropriate feedback or support based on their emotional needs [72]. Moreover, chatbots can be designed to express empathy through carefully crafted responses that acknowledge learners' feelings and offer encouragement [73]. By incorporating these techniques, chatbots can create a more emotionally supportive learning environment that fosters positive learner emotions and enhances engagement.

Moreover, to mitigate the lack of cultural context in chatbot-based language learning, it is crucial to design chatbots with culturally-sensitive and context-aware features. This involves incorporating cultural knowledge, norms, and values into the chatbot's knowledge base and conversation patterns [55]. By exposing learners to culturally authentic materials and scenarios, chatbots can help bridge the gap between language acquisition and real-world communication [74]. Additionally, chatbots can be programmed to recognize and respond appropriately to cultural references, idiomatic expressions, and social cues [75]. Designers can also consider creating chatbots with localized content and features that cater to specific cultural contexts and learner backgrounds [76]. By prioritizing cultural sensitivity and context-awareness, chatbots can provide a more immersive and authentic language learning experience that prepares learners for real-life interactions.

Furthermore, while AI-based chatbots offer numerous benefits, it is essential to integrate them with human-led instruction and peer collaboration to optimize language learning outcomes. Chatbots should be viewed as a complementary tool rather than a replacement for human teachers [77]. By combining chatbot-based practice with teacher-guided lessons and feedback, learners can benefit from both the personalized support of chatbots and the expertise and emotional connection of human instructors [78]. Moreover, incorporating peer collaboration activities alongside chatbot interactions can foster authentic communication skills and social learning [79]. For example, learners can engage in group discussions or collaborative projects, using chatbots as a resource for language support and feedback. This integration of human-led instruction, peer collaboration, and chatbot technology can create a comprehensive and emotionally engaging learning environment that caters to diverse learner needs.

Additionally, to address the ethical concerns and data privacy issues associated with AI-based chatbots in language education, it is crucial to establish clear ethical guidelines and data protection measures. Educational institutions and chatbot developers must prioritize learners' privacy and ensure that their personal information is collected, stored, and used responsibly [80]. This involves implementing secure data encryption, anonymization techniques, and strict access controls to prevent unauthorized use or disclosure of learner data [81]. Moreover, ethical guidelines should be developed to ensure that chatbots are designed and deployed in a manner that promotes fairness, transparency, and accountability [82]. This includes regularly auditing chatbot algorithms for biases and stereotypes, providing learners with clear information about how their data is used, and offering mechanisms for learners to provide feedback and report concerns [83]. By establishing robust ethical frameworks and data protection measures, educational institutions can foster trust and create a safe and inclusive learning environment for all learners.

As the field of AI-based language education continues to evolve, it is crucial to prioritize learner emotions in the design and implementation of chatbots. By creating emotionally supportive, culturally relevant, and ethically sound chatbot experiences, we can unlock the full potential of this technology to transform language learning. Future research should focus on developing more advanced affective computing techniques, exploring the long-term impact of chatbots on learner emotions and language acquisition, and investigating best practices for integrating chatbots into diverse educational contexts.

What's more, collaboration among researchers, educators, developers, and learners is essential for advancing the field and ensuring that chatbots meet the emotional and educational needs of language learners worldwide. By fostering interdisciplinary partnerships and engaging in ongoing dialogue, we can collectively work towards creating chatbot-based language learning experiences that are emotionally engaging, culturally responsive, and pedagogically effective. As we embrace the promises and navigate the challenges of AI-based chatbots in language education, let us keep learner emotions at the forefront of our efforts, striving to create a future where technology and empathy go hand in hand.

## 4 Future research

There are many research gaps in the literature, including AI digital literacy for teachers and students, chatbot-assisted learning behaviors and learning strategies etc [84]. These gaps can be examined in conjunction with learner emotions. For example, how does students' AI digital literacy affect students' positive and negative emotions such as enjoyment, boredom, anxiety, self-efficacy, and grit etc.? How do students' emotions (enjoyment, boredom, and grit etc.) affect chatbot-assisted language learning strategies? In addition, future research should focus on developing and validating new scales specifically designed to measure learner emotions in the context of using chatbots for language learning. While there are existing scales for measuring emotions in general educational settings, the unique nature of chatbot-based language learning requires tailored instruments. These scales should encompass a wide range of emotions, including positive emotions such as enjoyment, curiosity, and pride, as well as negative emotions like frustration, anxiety, and boredom (see [85]). Researchers should employ rigorous scale development procedures, such as exploratory and confirmatory factor analyses, to ensure the reliability and validity of these instruments [86]. By creating robust scales for assessing learner emotions in chatbot-based language learning, researchers can gain deeper insights into the emotional dynamics of these interactions and inform the design of emotionally intelligent chatbots.

To gain a comprehensive understanding of the emotional impact of chatbots on language learners, future research should conduct longitudinal studies. While cross-sectional studies provide valuable insights, longitudinal designs can reveal the long-term effects of chatbot interactions on learner emotions and language acquisition [87]. By collecting data at multiple points over an extended period, researchers can investigate how learner emotions evolve as they engage with chatbots and how these emotional experiences influence their language learning outcomes. Longitudinal studies can also shed light on the potential cumulative effects of chatbot-based learning on learner motivation, self-efficacy, and emotional well-being. These findings can inform the development of chatbots that provide sustained emotional support and foster long-term language learning success. Furthermore, future research should employ mixed-methods approaches to collect diverse data on the factors influencing and impacts of chatbots on language learners' emotions. By combining quantitative and qualitative methods, researchers can gain a more comprehensive and nuanced understanding of learner emotions in chatbot-based language learning. Quantitative methods, such as surveys and log data analysis, can provide insights into the prevalence and patterns of learner emotions, while qualitative methods, such as interviews and focus groups, can offer rich, in-depth accounts of learners' emotional experiences [88]. Moreover, collecting data from multiple sources, including learners, teachers, and chatbot developers, can provide a holistic perspective on the emotional dynamics of chatbot-learner interactions. By triangulating findings from diverse data sources and methods, researchers can identify key factors that influence learner emotions and develop strategies for optimizing chatbot design and implementation. Moreover, future research should conduct comparative analyses of different chatbot designs and their effects on learner emotions. As chatbot technologies continue to evolve, it is crucial to investigate how various design features, such as conversational styles, personalization strategies, and feedback mechanisms, influence learner emotions [89]. Researchers can conduct controlled experiments or quasi-experimental studies to compare the emotional impact of different chatbot designs on language learners. For example, studies can examine how learners' emotions differ when interacting with chatbots that employ empathetic versus neutral language, or chatbots that provide immediate versus delayed feedback [76]. By identifying the design elements that foster positive emotions and mitigate negative ones, researchers can inform the development of emotionally optimized chatbots for language learning. In addition, future research should explore the potential of chatbots in fostering emotional intelligence and intercultural competence among language learners. As language learning involves navigating complex emotional and cultural landscapes, chatbots that can support learners' emotional and intercultural development are highly valuable [90]. Researchers can investigate how chatbots can be designed to promote emotional self-awareness, empathy, and effective communication skills [91]. For example, chatbots can incorporate scenarios and prompts that encourage learners to reflect on their emotions and practice expressing them appropriately in the target language [92]. Additionally, researchers can examine how chatbots can be leveraged to foster intercultural competence by exposing learners to diverse cultural perspectives, norms, and practices [93]. By investigating the role of chatbots in supporting emotional intelligence and intercultural competence, researchers can contribute to the development of holistic language learning experiences that prepare learners for effective communication in a globalized world. Last but not least, future research should investigate the complex relationships among chatbots, learner emotions, and various individual and contextual factors. Language learners bring diverse backgrounds, personalities, and learning styles to their interactions with chatbots, which can influence their emotional experiences [94]. Researchers should examine how factors such as learners' age, gender, cultural background, language proficiency, and technology readiness impact their emotional responses to chatbot-based learning [95]. Moreover, contextual factors, such as the learning environment, task complexity, and social support, can also shape learners' emotions in chatbot interactions [96]. By examining the interplay among these variables, researchers can develop a more nuanced understanding of the emotional dynamics in chatbot-based language learning and inform the design of adaptive, emotionally intelligent chatbots that cater to diverse learner needs and contexts.

## 5 Conclusion

This conceptual analysis article has provided a comprehensive overview of the promises and challenges of AI-based chatbots in language education, with a particular focus on learner emotions. By integrating research from AI chatbots, positive psychology and language education, the paper has highlighted the crucial role of emotions in shaping learners' experiences and outcomes in chatbot-assisted language learning. The article has discussed the theoretical foundations underpinning the intersection of these two fields, emphasizing the need for a more holistic approach to understanding and optimizing chatbot-learner interactions. Moreover, the paper has explored the various scales used to measure learner emotions in chatbot-based language learning, as well as the factors, such as AI literacy, that influence these emotions. The article has also examined the promises of chatbots, such as personalized learning and increased motivation, and the challenges, including limited emotional intelligence and ethical concerns. Furthermore, the paper has proposed strategies for addressing these challenges and optimizing chatbot-learner interactions, such as incorporating affective computing techniques and designing culturally-sensitive chatbots. Finally, the article has outlined future research directions, emphasizing the need for validated emotion scales, longitudinal studies, mixed-methods approaches, comparative analyses, and investigations into the role of chatbots in fostering emotional intelligence and intercultural competence. Based on the insights gained from this article, several practical recommendations can be made for educators, researchers, and chatbot developers. Educators should strive to integrate chatbots into their language teaching practices in a way that prioritizes learner emotions and fosters a supportive, engaging learning environment. This can involve selecting chatbots that offer personalized feedback, culturally-relevant content, and emotionally intelligent interactions. Educators should also provide learners with guidance on how to effectively use chatbots and encourage them to reflect on their emotional experiences during chatbot-assisted learning. Researchers should continue to investigate the complex relationships among chatbots, learner emotions, and various individual and contextual factors, employing diverse methodologies and collaborating across disciplines. They should also work towards developing and validating emotion scales specific to chatbot-based language learning and conducting longitudinal studies to understand the long-term emotional impact of chatbots. Chatbot developers should prioritize the incorporation of affective computing techniques, culturally-sensitive features, and ethical design principles in their creations. They should collaborate closely with educators and researchers to ensure that their chatbots align with pedagogical goals and learner needs, and continuously iterate based on user feedback and emerging research insights. As this conceptual analysis review article has demonstrated, learner emotions play a pivotal role in the success and effectiveness of AI-based chatbot assisted language learning and vice versa. Emotions influence learners' motivation, engagement, and overall language acquisition outcomes, and thus cannot be overlooked in the design, implementation, and evaluation of chatbot technologies. By prioritizing learner emotions, educators, researchers, and developers can create chatbot-based language learning experiences that are not only cognitively stimulating but also emotionally supportive and empowering. This holistic approach to chatbot-assisted language education has the potential to transform the way learners acquire languages, fostering a more positive, inclusive, and emotionally intelligent learning environment. As the field continues to evolve, it is crucial for all stakeholders to keep learner emotions at the forefront of their efforts, striving to harness the power of AI-based chatbots to create truly transformative language learning experiences. By doing so, we can unlock the full potential of this innovative technology and support learners in their journeys towards linguistic proficiency and personal growth.

## Data availability statement

No data were used for the research described in this conceptual analysis review article.

## Ethics statement

The authors followed ethical guidelines stated in Elsevier's Publishing Ethics Policy.

As this is a review paper, no human participants were involved in this research to provide empirical data.

## Funding

This study was funded by the National Social Sciences Fund of China for Chinese Scholarly Works Translation (grant number: 20WYYA002).

## CRediT authorship contribution statement

**Yuehai Xiao:** Writing – review & editing, Writing – original draft, Resources, Methodology, Investigation, Funding acquisition, Conceptualization. **Tianyu Zhang:** Writing – review & editing, Writing – original draft. **Jingyi He:** Writing – review & editing.

## Declaration of competing interest

There are no identified conflicts of interest, financial or otherwise, nor are there personal connections that could be perceived as having affected this review paper.
